# Clinical Effect of Emergency Dermabrasion Combined with Biological Dressing A on Wound Microcirculation and Preventing Sepsis in Deep Degree-II Burns

**DOI:** 10.1155/2022/4730905

**Published:** 2022-07-14

**Authors:** Huawei Shao, Ru Luo, Chuangang You, Qiong Li, Shulei Mao

**Affiliations:** ^1^Department of Burns & Wound Care Centre, 2nd Affiliated Hospital of Zhejiang University, College of Medicine, Hangzhou, Zhejiang 310030, China; ^2^Department of Pathology, 2nd Affiliated Hospital of Zhejiang University, College of Medicine, Hangzhou, Zhejiang 310030, China; ^3^Department of Burns and Plastic Surgery, Zhejiang Quhua Hospital, Quzhou, Zhejiang 324004, China

## Abstract

**Objective:**

The aim of this study is to explore the clinical effect of emergency dermabrasion combined with biological dressing A on wound microcirculation and preventing sepsis in deep degree-II burns.

**Methods:**

A total of 90 patients with deep degree-II burns admitted to the hospital were retrospectively enrolled between January 2020 and January 2022. According to different treatment methods, they were divided into the control group (42 cases, biological dressing A) and the observation group (48 cases, emergency dermabrasion combined with biological dressing A). The clinical curative effect in both groups was observed. The wound repair rate and wound healing quality, and changes in levels of wound microcirculation-related indexes (serum epidermal growth factor (EGF), wound blood flow, and partial pressure of transcutaneous oxygen) and inflammatory cytokines (C-reactive protein (CPR), interleukin-6 (IL-6), erythrocyte sedimentation rate (ESR), and procalcitonin (PCT)) before treatment, at 3d and 7d after treatment were compared between the two groups. The incidence of wound infection and sepsis in both groups was recorded.

**Results:**

The wound healing time in the observation group was significantly shorter than that in the control group, and wound healing quality in the observation group was better than that in the control group (*P* < 0.05). At 3 d and 7d after treatment, the levels of serum EGF, wound blood flow and partial pressure of transcutaneous oxygen in both groups were all increased (*P* < 0.05), which were higher in the observation group than those in the control group (*P* < 0.05). The levels of CRP, IL-6, ESR, and PCT in both groups were all decreased (*P* < 0.05), which were lower in the observation group than those in the control group (*P* < 0.05). There was no significant difference in incidence of sepsis between observation group and control group (4.17% (2/48) vs. 7.14% (3/42)) (*Fisher* = 0.539).

**Conclusion:**

Emergency dermabrasion combined with biological dressing A can effectively improve wound microcirculation in patients with deep degree-II burns, promote wound healing, shorten wound healing time, improve wound healing quality, effectively control inflammatory response, and prevent sepsis.

## 1. Introduction

The skin plays an important role in protecting and regulating the body and plays an important role in promoting the body's metabolism and maintaining internal stability. Burn refers to the tissue damage caused by the contact of skin tissue with heat, which is a common traumatic disease in surgery [1]. According to the depth of the burn, the clinical treatment plan is also different. For patients with superficial burns, the skin still has the self-healing function that can be healed within 2 weeks and the clinical symptoms are mainly relieved. For patients with deep burns, because the dermis has been damaged, the dermis cannot be regenerated below the papillary layer; the burn wound is difficult to heal and the healing process is easy to be infected [2], which is unfavorable for their prognosis. Therefore, it is of great clinical significance to improve the wound healing efficiency and improve the quality of wound healing in clinical deep burn patients. Biological dressing A is a commonly used dressing in clinical practice. Its raw material is mainly porcine collagen, which is rich in fibrin, skin trace elements, etc., which can effectively maintain the electrolyte balance of the wound and promote wound healing [3]. Its significance is the most concerned operation of therapeutic care and can be effectively used to treat tissue, care for important parts, and help wounds heal [4]. In order to further understand its application effect in patients with deep burns, this study conducted a retrospective analysis of deep second-degree burns treated in our hospital, which provided clinical supplementary evidence-based basis.

## 2. Materials and Methods

### 2.1. General Information

A total of 90 patients with deep second-degree burns who were admitted to our hospital from January 2020 to January 2022 were retrospectively selected and divided into the control group (42 cases) and the observation group (48 cases) according to their treatment plan.

In the observation group, there were 25 males and 23 female. The age ranged from 23 to 47 years old, with an average age of (33.88 ± 5.40) years old; the average burn area was (37.33 ± 3.07)%. Burn sites: 22 cases of head and face, 19 cases of limbs, and 7 cases of trunk. Causes of burns: liquid burns in 20 cases, chemical burns in 15 cases, and flame burns in 13 cases.

The control group consisted of 21 males and 24 females; The age ranged from 24 to 47 years old, with an average age of (35.14 ± 5.13) years old. The average burn area was (37.93 ± 3.34)%. Burn sites: 17 cases of head and face, 19 cases of limbs, and 6 cases of trunk. Causes of burns: liquid burns in 17 cases, chemical burns in 12 cases, and flame burns in 13 cases. There was no difference in the clinical baseline data between the two groups (*P* > 0.05) and a comparison between the two groups was feasible.

The inclusion criteria were as follows: ① those who were diagnosed with deep second-degree burns [5]; ② those who were admitted to the hospital within 48 hours after the burn and there was local infection of the wound; ③ no third-degree and above burns were found. The exclusion criteria were as follows: ① those with severe shock at the time of admission; ② patients with systemic infection or combined with malignant tumor at the time of admission; ③ those with moderate to severe inhalation injury; ④ those with chronic diseases such as diabetes or coronary heart disease before; ⑤ there are long-term immunosuppressive or hormonal drug users; ⑥ superficial burns (first degree or superficial second degree burns); and ⑦ women who are pregnant or breastfeeding.

### 2.2. Methods

Both groups received basic treatments such as routine wound debridement, maintenance of electrolyte balance, and pit infection.

The wounds of patients in the control group were treated with biological dressing A: Biological dressing A was collected from Shandong Weihai Huate Biotechnology Co., Ltd. and used pig collagen as the main raw material. After routine debridement and rotten skin removal, a sterile biological dressing A larger than 5 cm from the wound edge was cut and applied to the debridement surface. The layer dressing was changed, then we were waiting for the dressing to be closely attached to the wound, and the scab will naturally dry and fall off.

On the basis of the control group, patients in the observation group were combined with emergency escharectomy. When the patients were admitted to the hospital, emergency escharectomy was performed. According to the patient's condition, an appropriate anesthesia method was chosen. After the anesthesia effect takes effect, routine burn wound disinfection is performed. Rub the wound with a steel ball, grind it carefully, and grind the teeth with industrial sand. All scabs were removed, and the wound appeared pale and necrotic, with uniform and dense small bleeding points. After that, the friction was stopped and the wound was rinsed with sterile normal saline. After repeated washing, the wound was wet compressed with amikacin saline for at least 5 min. Then, the sterile biological dressing A larger than 5 cm from the wound edge was cut and applied to the eschar wound. The outside is covered with a gauze and bandage (thickness 3∼5 cm), and the outer dressing is changed every 2∼3 days, waiting for the dressing and the wound to apply closely, dry, and scab off naturally.

### 2.3. Indicators

1. In both groups, the wound repair status after 3 months of wound treatment was used as the evaluation of clinical efficacy. The wound repair rate and wound healing quality of the two groups of patients were compared: Wound healing standard: the basal epithelialization of the wound was ≥95%, and there was no exudate on the wound surface, and no outer dressing was required for the process of bandaging and fixation. Wound quality was assessed using the Vancouver Scar Scale (VSS) [6]. The VSS scale includes skin color, thickness, vascularity, and flexibility, with a total score of 15 points. The higher the score, the worse the wound recovery.
2. Comparison of wound microcirculation-related indicators (serum epidermal growth factor (EGF), wound blood flow and transcutaneous partial pressure of oxygen (TcpO2)) and inflammatory cytokines (C-reactive protein (CPR), interleukin-6 (IL-6), erythrocyte sedimentation rate (ESR), and calcitonin (PCT)) levels. EGF, CPR, IL-6, and PCT adopt the enzyme-linked adsorption method, and the kits are all from Shanghai Qiyan Biotechnology Co., Ltd., and the ESR adopts an automatic biochemical analyzer (Beckman AU5800). All operations were carried out by the laboratory department of our hospital in strict accordance with the kit instructions. Wound blood flow and percutaneous oxygen partial pressure were detected by a color Doppler perfusion imager (Bessman BV-520T).
3. The incidence of wound infection and sepsis within 3 months after wound treatment in the two groups was recorded.

### 2.4. Statistical Processing

The database of this scientific research project was constructed, and the statistical software SPSS 22.0 was used to complete the statistical processing of the data of this scientific research project. The Shapiro–Wilk test method was used to test the normality of the measurement data, and the measurement data that met the normal distribution and the variance were expressed as ($\bar{x}\pm s$). Differences between the two groups were compared using an independent *t*-test. Differences within groups were compared using paired *t*-test. We infer whether the population means represented by two or more sample means are different using one-way ANOVA. The enumeration data were expressed as rates, and the *χ*2 test or Fisher's exact test was used. *P* < 0.05 indicated that the difference was statistically significant.

## 3. Results

### 3.1. Illustration of Typical Cases before and after Treatment

#### 3.1.1. Case Illustration of Emergency Escharectomy Combined with Biological Dressing A

Figures 1–3 show a 47-year-old male patient who was admitted to the hospital due to multiple hot iron scalds all over the body.  Figure 1 shows the performance before treatment.  Figure 2 shows the 3d performance after treatment.  Figure 3 shows the performance 7d after treatment.

#### 3.1.2. Illustration of the Case of Using Biological Dressing A Alone

Figures 4–6 show a 25-year-old male patient who was admitted to the hospital due to hot oil flame burns on both upper extremities. After cleaning, the biological dressing A was directly applied.  Figure 4 shows the performance before treatment.  Figure 5 shows the performance 3d after treatment.  Figure 6 shows the performance 7d after treatment.

### 3.2. Comparison of the Wound Healing Rate and Wound Healing Quality between the Two Groups of Patients

The wound healing time in the observation group was shorter than that in the control group, and the wound healing quality in the observation group was better than that in the control group (*P* < 0.05) as shown in Figure 7.

### 3.3. Comparison of Wound Microcirculation before and after Treatment between the Two Groups of Patients

At 3d and 7d after treatment, the serum EGF level, wound blood flow, and TcpO2 index increased in both groups (*P* < 0.05) and those of the observation group wereas more significant (*P* < 0.05) as shown in Figures 8–10.

### 3.4. Comparison of Inflammatory Factor Levels before and after Treatment in the Two Groups of Patients

At 3d and 7d after treatment, the levels of CRP, IL-6, ESR, PCT, and other inflammatory indexes in the two groups were decreased (*P* < 0.05) and those of the observation group were more significant (*P* < 0.05) as shown in Figures 11–14.

### 3.5. Comparison of the Incidence of Wound Infection and Sepsis between the Two Groups of Patients

The incidence of sepsis in the observation group was 4.17% (2/48) compared with 7.14% (3/42) in the control group, which had no significant difference (Fisher = 0.539).

## 4. Discussions

Deep second-degree burns have damaged the dermis layer, the wound heals slowly and may leave large scars, which is not conducive to the recovery of skin function and affects the prognosis [7]. Thus, it is very important to improve the quality of wound healing in patients. Biological dressing A is rich in fibrils and mucins, has good wound adhesion, and can provide a good environment for wound healing. It is a commonly used clinical wound dressing. Escharectomy is a wound treatment method that has received high clinical attention in recent years. It can effectively clean up the necrotic tissue on the wound surface and create a good foundation for subsequent operations, thereby improving the clinical effect and effectively improving the quality of wound healing [8, 9]. This study retrospectively analyzed the application effect of emergency escharectomy combined with biological dressing A, which provided clinical supplementary evidence-based basis.

The results of our study showed that the wound healing time in the observation group was shorter than that in the control group, and the wound healing quality in the observation group was better than that in the control group. It is suggested that the combined application of emergency escharectomy and biological dressing A can effectively improve the wound healing effect. The reason may be that scab rubbing uses a medical friction ball to treat the wound surface with mild force, which has a certain protective effect on the normal tissue around the wound surface [9], avoiding secondary damage, and it should be compared with traditional debridement. Due to the smaller shock response, the quality of subsequent recovery is better. EGF is an active substance in the blood, which can stimulate the growth factor of epidermal cells, promote the repair and regeneration of damaged skin, and accelerate wound healing [10]. Both the wound blood flow and the transdermal oxygen pressure index reflect the An indicator of wound blood flow status. The study showed that 3d and 7d after treatment, the serum EGF level, wound blood flow, and transcutaneous oxygen partial pressure index increased in both groups, especially in the observation group. This result suggests that the treatment regimens of both groups can effectively improve the microcirculation of burn wounds, but the effect of the observation group is better. Analysis of the reason may be that escharectomy also has a massage and dredging effect on the wound stasis belt during the operation, which can effectively improve the blood state of the surface tissue of the wound skin, promote the blood circulation of the wound, and improve the microcirculation of the wound [11], thereby increasing serum EGF levels and promoting wound repair, and it is also a major reason for the shortened wound healing time.

The occurrence of sepsis is closely related to the prognosis of patients, so clinical attention is paid to reduce the incidence of sepsis. CRP is an acute phase reaction protein, and its level increases when the body is infected. It is a routine indicator for clinical detection of inflammation; the change in the IL-6 level is an important indicator to reflect the degree of inflammation in the body [12]. ESR refers to the rate of red blood cell deposition, and its level increases in the event of trauma and infection [13]. PCT has a high specificity in sepsis [14]. The study showed that the levels of CRP, IL-6, ESR, PCT, and other inflammatory indicators decreased in the two groups at 3d and 7d after treatment, among which the observation group was more to be significant. Analysis of the reason may be that escharectomy can improve the blood flow state of the wound, increase the permeability, and effectively reduce the inflammatory response, which was also reflected in an animal study [15]. Biological dressing A has a high degree of adhesion to the wound surface and can effectively isolate the wound surface from contact with the external environment. The combination of the two can effectively reduce the inflammatory response of the wound surface [16]. There was no difference in the incidence of sepsis between the two groups, suggesting that both schemes are effective in the prevention of sepsis. However, because the development of sepsis is related to wound infection, it is believed that emergency dermabrasion combined with biological dressing A is effective for sepsis. Disease prevention is more dominant.

In conclusion, emergency escharectomy combined with biological dressing can effectively improve deep II degree burns, can make the patient's wound microcirculation, promote wound healing, continuous burn wound time, and improve the quality of surface healing, and it can effectively control the inflammatory response and fail to acupuncture.

## Figures and Tables

**Figure 1:** Prior treatment.

**Figure 2:** 3d after treatment.

**Figure 3:** 7d after treatment.

**Figure 4:** Prior treatment.

**Figure 5:** 3d after treatment.

**Figure 6:** 7d after treatment.

**Figure 7:** Comparison of wound repair rate and wound healing quality between the two groups.

**Figure 8:** Comparison of EGR between the two groups before and after treatment.

**Figure 9:** Comparison of wound blood flow between the two groups before and after treatment.

**Figure 10:** Comparison of TcpO_2_ between the two groups before and after treatment.

**Figure 11:** Comparison of CRP between the two groups before and after treatment.

**Figure 12:** Comparison of IL-6 between the two groups before and after treatment.

**Figure 13:** Comparison of ESR between the two groups before and after treatment.

**Figure 14:** Comparison of PCT between the two groups before and after treatment.

## Data Availability

The data used and/or analyzed during the current study are available from the corresponding author upon request.
